# Effect of Admission Serum Calcium Levels and Length of Stay in Patients with Acute Pancreatitis: Data from the MIMIC-III Database

**DOI:** 10.1155/2022/4275283

**Published:** 2022-06-20

**Authors:** Dongyan Wang, Xiaoyan Guo, Wenwen Xia, Zhijuan Ru, Yihai Shi, Zhengyu Hu

**Affiliations:** ^1^Department of Gastroenterology, Shanghai Pudong New Area Gongli Hospital, Shanghai 200135, China; ^2^Department of Gastroenterology, Shanghai Tenth People's Hospital, Tongji University School of Medicine, Shanghai 200072, China; ^3^Department of General Surgery, Shanghai Tenth People's Hospital, Tongji University School of Medicine, Shanghai 200072, China

## Abstract

**Objective:**

We retrospectively investigated the effect of admission serum calcium levels on length of stay (LOS) in patients hospitalized with acute pancreatitis (AP).

**Methods:**

Clinical data for 3156 patients diagnosed with AP were obtained from the Multiparametric Intelligent Monitoring in Intensive Care III (MIMIC-III) database. Restricted cubic spline curve (RCS) functions of dose-response analysis curves and logistic regression analysis were used to analyze the relationship between admission serum calcium levels and the LOS.

**Results:**

All patients were divided into 2 groups (<8.5 mg/dl group and ≥8.5 mg/dl group) based on RCS analysis. RCS showed a significant nonlinear negative correlation between blood calcium levels and the LOS (*p* < 0.001). In addition, compared with patients with blood calcium <8.5 mg/dl, multivariate logistic regression analysis showed that patients with blood calcium ≥8.5 mg/dl had a reduced risk of the LOS >2 days (aOR = 0.653; 95% CI 0.507–0.842; *p*=0.001), a reduced risk of the LOS >5 days (aOR = 0.589; 95% CI 0.503–0.689; *p* < 0.001), and a reduced risk of the LOS >7 days (aOR = 0.515; 95% CI 0.437–0.609; *p* < 0.001). And similar results were found in the subgroup analysis.

**Conclusion:**

Our findings suggest that low blood calcium increases the LOS in patients with AP. More attention is needed for patients with combined low blood calcium levels (<8.5 mg/dl) in hospitalized AP patients.

## 1. Introduction

Acute pancreatitis (AP) is an autodigestive disease of the pancreas resulting from abnormal activation of pancreatic enzymes due to multiple etiologies, of which approximately 20% of patients may develop severe acute pancreatitis (SAP) [1]. Attributed to hyperlipidemia, cholelithiasis, smoking, alcohol consumption, diabetes, and obesity, the incidence of SAP is increasing year by year and increases the overall economic burden on the public health system [2, 3].

Pancreatitis is common in the United States and affects 40/100,000 people per year, resulting in more than 300,000 hospitalizations and 20,000 deaths each year at a cost of more than $2.2 billion per year [4]. Multiple studies have shown that aberrant regulation of Ca^2+^ signaling is a key trigger in the pathogenesis of AP [5, 6]. The incidence of hypocalcemia is significantly higher in patients with SAP than in those with mild AP. In addition, a significant negative correlation between the incidence of sepsis and the serum calcium concentration was observed [7].

Calcium, as the most abundant mineral in the body, has many essential functions, including muscle function, neurotransmission, intracellular signaling, and mediating vasoconstriction and vasodilation [8, 9]. Several retrospective studies have demonstrated the impact of serum calcium levels on adverse clinical outcomes, including in-hospital all-cause mortality, complications, and increased length of stay (LOS) [10–12]. Nevertheless, the relationship between serum calcium levels and the LOS in AP patients is still unclear. In this study, we analyzed the influence of serum calcium levels on the LOS of patients with AP and its possible influencing factors.

## 2. Patients and Methods

### 2.1. Study Design and Data Retrieval

Subject data of AP patients were retrieved using Structured Query Language (SQL) software from the Multiparameter Intelligent Monitoring in Intensive Care III (MIMIC-III) database version 1.4, a multiparameter critical care database developed by the Massachusetts Institute of Technology. The database opened to the public and included demographic data, medical intervention records, basic physical signs, nursing records, imaging findings, and discharge records of over 40,000 adult intensive care unit (ICU) stays admitted to the Beth Israel Deaconess Medical Center (BIDMC) in the United States from 2001 to 2012 [13]. After completing a network training course at the National Institute for the Study of Human Health Protection, we were granted permission to extract data from the MIMIC-III database (certification number. 44292607). This study was an analysis of a public database that did not require informed patient consent and institutional review board approval as all data associated with patient identification information were multiply encrypted.

We excluded patients with (1) lacking serum calcium information within 24 hours of admission (*n* = 676); (2) less than 24 hours of hospitalization (*n* = 249). Eventually, 3156 people were included (Figure 1).

### 2.2. Population Selection and Covariates

According to the International Classification of Diseases, ninth revision (ICD-9, code 577.0) and tenth revision (ICD-10, code K85), we obtained the hadm id identifiers of 4081 patients (age ≥18 years) diagnosed with AP from the MIMIC-III database. We extracted information about demographic information, comorbidities, laboratory tests, length of hospitalization, and hospital death. Demographic information included age, gender, ethnicity, marital status, and insurance status. Comorbidity information included chronic heart failure (CHF), hypertension, chronic obstructive pulmonary disease (COPD), diabetes mellitus, renal failure, liver disease, coronary artery disease (CAD), hyperlipidemia, admission to the intensive care unit (ICU), Charlson comorbidity index (CCI), sequential organ failure assessment (SOFA) score, systemic inflammatory response system (SIRS) score, and simplified acute physiology score II (SAPSII) score. Laboratory tests included white blood cell count, albumin, total bilirubin (TBil), lipase, amylase, aspartate aminotransferase (AST), alanine aminotransferase (ALT), blood urea nitrogen (BUN), creatinine, and glucose.

### 2.3. Statistical Analysis

Continuous variables were expressed as the median and interquartile range (IQR) while categorical ones as frequency (*n*, %). For categorical variables, we used *χ*^2^ test for comparison between the groups. The Kruskal–Wallis test was used in the nonnormal model to assess continuous variables. The LOS was regarded as a dichotomized variable (≤2 days or >2 days, ≤5 days or >5 days, and ≤7 days or >7 days). The restricted cubic spline (RCS) model can fit the dose-response relationship between continuous variables and outcomes more intuitively. The RCS model was used to confirm the association between serum calcium levels and the LOS >2 days, LOS >5 days, or LOS >7 days. The relationship between serum calcium levels and the LOS >2 days, LOS >5 days, or LOS >7 days was assessed using univariate and multivariate logistic regression methods, and adjusted odds ratios (aORs) and 95% confidence intervals (CIs) were calculated. We constructed three distinct models in multivariate logistic regression analysis. Model A included five variables from the demographic information. Model B included the variables from model A and thirteen variables from the comorbidity information, and model C included the variables from model B and nine variables from the laboratory test information. In addition, we performed the same analysis for subgroups with a proportion greater than 50% to determine the relationship between serum calcium levels and the LOS in the subgroups.

SPSS software (version 24.0) and RStudio software (version 1.4.1106) were used for all statistical analyses in this study. A *p* value <0.05 was considered statistically significant by a two-tailed test.

## 3. Results

The final study included data from 3156 patients. After correction for demographic variables, comorbidity variables, and variables in laboratory tests, the RCS dose-response curves showed a significant nonlinear negative correlation between blood calcium levels and the LOS >2 days, LOS >5 days, and LOS >7 days (all *p* < 0.001) (Figure 2).

In the RCS model, we calculated the blood calcium concentration at aOR = 1 to be 8.5 mg/dl (approximately 2.125 mmol/L). We then divided all AP patients into 2 groups: a low blood calcium group (<8.5 mg/dl) and a high blood calcium group (≥8.5 mg/dl). We compared the demographic and clinic pathologic characteristics of patients in the two groups and found differences in race, insurance, CAD, hyperlipidemia, admission to the ICU, WBC, albumin, TBil, AST, BUN, glucose, bicarbonate, sodium, potassium, LOS, and in-hospital mortality (Table 1). The serum calcium <8.5 mg/dl group had a higher percentage of other races (20.9%), Medicare (35.1%), Medicaid (11.5%) coverage, without CAD (88.1%), without hyperlipidemia (75.3%), and ICU admission (23.7%). Compared to the serum calcium ≥8.5 mg/dl group, patients in the serum calcium <8.5 mg/dl group had higher levels of WBC [9.40(6.50, 13.90) 10^9^/L], TBil [1.00(0.50, 2.40) mmol/L], AST [65.0(29.0, 145.0) U/L], BUN [14.0(9.0, 22.0) mmol/L ], blood glucose [106.0 (87.0, 139.0) mg/dL] and lower levels of albumin [3.10 (2.70, 3.50) g/L], bicarbonate [24.0 (21.0, 26.0) mmol/L], sodium [139.0 (136.0, 141.0) mmol/L], and potassium [3.90 (3.50, 4.20) mmol/L]. In addition, the serum calcium <8.5 mg/dl group had a higher in-hospital mortality rate (5.3%) and a longer hospital stay [5.81(3.43, 11.49) days].

We used logistic regression analysis to assess the relationship between serum calcium levels and the LOS. Univariate analysis showed a significantly lower risk of LOS >2 days, LOS >5 days, and LOS >7 days in the group with blood calcium levels ≥8.5 mg/dl compared with the group with blood calcium levels <8.5 mg/dl. In addition, compared with patients with blood calcium <8.5 mg/dl, multivariate logistic regression analysis showed that patients with blood calcium ≥8.5 mg/dl had a reduced risk of LOS >2 days (aOR = 0.653; 95% CI 0.507–0.842; *p*=0.001), a reduced risk of LOS >5 days (aOR = 0.589; 95% CI 0.503–0.689; *p* < 0.001), and a reduced risk of LOS >7 days (aOR = 0.515; 95% CI 0.437–0.609; *p* < 0.001) (Table 2).

We obtained similar results in the subgroup analysis. In a subgroup logistic regression analysis of males, age <60 years, white, without CHF, without hypertension, without diabetes, without renal failure, without liver disease, without coronary artery disease, without hyperlipidemia, and non-ICU admissions, we found that the serum calcium level ≥8.5 mg/dl patients had a lower risk for LOS >2 days (Figure 3), LOS >5 days (Figure 4), and LOS >7 days (Figure 5) than the serum calcium level <8.5 mg/dl patients in all subgroups.

## 4. Discussion

In this retrospective study, we investigated the relationship between serum calcium levels and the LOS by analyzing clinical data from 3156 AP inpatients in the MIMIC-III database using the RCS model and univariate and multivariate logistic regression analyses. Dose-response curve analysis of the RCS model showed a significant nonlinear negative relationship between serum calcium levels and the LOS >2 days, LOS >5 days, and LOS >7 days, with serum decrease in calcium levels significantly increasing the risk of LOS prolongation. In addition, multivariate logistic regression analysis showed that patients with blood calcium levels ≥8.5 mg/dl had a significantly lower risk of LOS >2 days, LOS >5 days, and LOS >7 days than patients with blood calcium levels <8.5 mg/dl.

As is known, the severity of AP ultimately depends on the intensity of the systemic inflammatory response [14]. The excessive inflammatory response is key to the multiorgan dysfunction associated with the course of SAP. Previous studies have shown a correlation between calcium clearance levels and the severity of AP [15, 16], and hypocalcemia has been included in the prognostic scoring system for AP [17]. Although the exact mechanism by which hypocalcemia occurs in AP is unknown, the vast majority of studies suggest that acute pancreatitis leads to the release of a large number of reactive enzymes in the pancreas, including lipase. Lipase breaks down fats in the pancreas and circulation-forming free fatty acids which bind to calcium ions to form insoluble particles, leading to hypocalcemia [18, 19]. In the study cohort, we also found that the median lipase level was higher in the low serum calcium group than in the serum calcium level ≥8.5 mg/dl group. Therefore, serum calcium levels are closely related to the inflammatory response during AP, hypocalcemia also predicts a state of severe damage to the pancreas, and hypocalcemia status can be used as one of the clinical reference indicators to assess the severity of AP [20, 21].

We used the RCS model to fit a cut-off value of serum calcium = 8.5 mg/dl for grouping and could find that patients with serum calcium <8.5 mg/dl had a significantly increased risk of prolonged LOS and in-hospital mortality. In recent years, a growing number of studies have found that serum calcium levels affect the LOS and all-cause mortality in hospitalized patients [11, 12, 22]. With the recent introduction of the concept of promoting recovery after surgery (ERAS) in the management of surgical diseases, it is generally accepted that, except for albumin or body mass index, calcium or phosphorus may also be important indicators for assessing the nutritional status of surgical patients [23, 24]. Decreased serum calcium is common in critically ill patients and correlates with the severity of the disease [24, 25]. In addition, serum calcium may be reduced after blood transfusion, plasma replacement, and parathyroidectomy [26–28]. In the present study, we performed a subgroup analysis after fully adjusting for all factors that may affect the LOS and found that a decrease in serum calcium (<8.5 mg/dL) during hospitalization was significantly associated with a prolongation of the LOS. Although the underlying mechanisms remain unclear, some studies suggest that a decrease in serum calcium can significantly alter myocardial action potential [29] and reduce renal sodium excretion [30], leading to circulating fluid overload and reduced myocardial contractility [31–33].

However, there are also some limitations of our study. Firstly, this retrospective cohort study was based on the MIMIC-III database, in which some clinical treatment information was missing (e.g., treatment of calcium disorder abnormalities, oral calcium supplements, and intravenous calcium infusion) thus not represented in this study. Secondly, despite our extensive adjustment for potential confounders, the association between serum calcium and the LOS may still be confounded by unmeasured confounders. Finally, our study does not provide effective conclusions to demonstrate that calcium supplementation in AP patients can reduce the risk of mortality, LOS, and hospitalization costs. This relies on further RCT studies.

## 5. Conclusions

In summary, we found that low serum calcium levels on admission were associated with prolonged LOS in admitted AP patients. Therefore, this group of patients should be taken more seriously and require a higher level of care.

## Figures and Tables

**Figure 1:** Schematic flow diagram of exclusion criteria for the study cohort.

**Figure 2:** Relative risk for a hospital length of stay (LOS) >2 days, >5 days, and >7 days according to the serum calcium level. The solid black lines represent aORs based on restricted cubic splines for the serum calcium level. The dotted curve represents upper and lower 95% CIs. Adjustment factors are the same as those in the extended model of Table 2.

**Figure 3:** Results of subgroup analyses of the serum calcium level and a hospital length of stay (LOS) >2 days according to clinical characteristics.

**Figure 4:** Results of subgroup analyses of the serum calcium level and a hospital length of stay (LOS) >5 days according to clinical characteristics.

**Figure 5:** Results of subgroup analyses of the serum calcium level and a hospital length of stay (LOS) >7 days according to clinical characteristics.

**Table 1:** Participants' baseline characteristics.

Characteristics		Serum calcium (mg/dl)				*p* value
		All patients no. (%)	Low serum calcium <8.5 no. (%)		High serum calcium ≥8.5 no. (%)	
Total patients		3156	1580 (50.1)		1576 (49.9)	
Demographics						
Age, years	58.32 (45.96, 71.75)		58.21 (45.92, 72.08)	58.47 (46.02, 71.27)		0.405
Age categorized, years						0.827
<60	1682 (53.3)		839 (53.1)	843 (53.5)		
≥60	1474 (46.7)		741 (46.9)	733 (46.5)		
Gender						0.434
Male	1600 (50.7)		812 (51.4)	788 (50.0)		
Female	1556 (49.3)		768 (48.6)	788 (50.0)		
Ethnicity						0.003
White	2185 (69.2)		1095 (69.3)	1090 (69.2)		
Black	362 (11.5)		155 (9.8)	207 (13.1)		
Others	609 (19.3)		330 (20.9)	279 (17.7)		
Marital status						0.588
Married	1439 (45.6)		728 (46.1)	711 (45.1)		
Nonmarried	1717 (54.4)		852 (53.9)	865 (54.9)		
Insurance						0.002
Medicare	1045 (31.1)		555 (35.1)	490 (31.1)		
Medicaid	332 (10.5)		182 (11.5)	150 (9.5)		
Others	1779 (56.4)		843 (53.4)	936 (59.4)		
Comorbidities						
CHF						0.671
No	2960 (93.8)		1479 (93.6)	1481 (94.0)		
Yes	196 (6.2)		101 (6.4)	95 (6.0)		
Hypertension						0.819
No	2239 (70.9)		1118 (70.8)	1121 (71.1)		
Yes	917 (29.1)		462 (29.2)	455 (28.9)		
COPD						0.640
No	3138 (99.4)		1570 (99.4)	1568 (99.5)		
Yes	18 (0.6)		10 (0.6)	8 (0.5)		
Diabetes mellitus						0.465
No	2626 (83.2)		1307 (82.7)	1319 (83.7)		
Yes	530 (16.8)		273 (17.3)	257 (16.3)		
Renal failure						0.541
No	3052 (96.7)		1531 (96.9)	1521 (96.5)		
Yes	104 (3.3)		49 (3.1)	55 (3.5)		
Liver disease						0.541
No	3052 (96.7)		1531 (96.9)	1521 (96.5)		
Yes	104 (3.3)		49 (3.1)	55 (3.5)		
CAD						0.029
No	2739 (86.8)		1392 (88.1)	1347 (85.5)		
Yes	417 (13.2)		188 (11.9)	229 (14.5)		
Hyperlipidemia						0.021
No	2318 (73.4)		1189 (75.3)	1129 (71.6)		
Yes	838 (26.6)		391 (24.7)	447 (28.4)		
Admitted to the ICU						<0.001
No	2663 (84.4)		1206 (76.3)	1457 (92.4)		
Yes	493 (15.6)		374 (23.7)	119 (7.6)		
CCI	4.0 (2.0, 6.0)		4.0 (2.0, 6.0)	4.0 (2.0, 6.0)		0.208
SOFA score	1.0 (0.0, 3.0)		1.0 (0.0, 3.0)	1.0 (0.0, 2.0)		0.347
SIRS score	3.0 (2.0, 4.0)		3.0 (3.0, 4.0)	3.0 (2.0, 3.0)		0.059
SAPSII score	38.0 (28.0, 50.0)		38.0 (28.0, 50.0)	36.0 (28.0, 48.0)		0.447
Lab examination						
WBC, 10^9^/L	8.85 (6.30, 12.60)		9.40 (6.50, 13.90)	8.30 (6.10, 11.50)		<0.001
Albumin, g/L	3.40 (2.90, 3.80)		3.10 (2.70, 3.50)	3.70 (3.30, 4.00)		<0.001
TBil, mmol/L	0.90 (0.50, 2.10)		1.00 (0.50, 2.40)	0.80 (0.50, 1.80)		<0.001
Lipase, IU/L	186.0 (61.0, 701.0)		198.0 (65.0, 721.0)	173.0 (57.8, 677.3)		0.259
Amylase, IU/L	148.0 (66.0, 410.0)		153.0 (65.5, 433.5)	144.0 (66.0, 402.5)		0.632
AST, U/L	57.0 (25.0, 142.0)		65.0 (29.0, 145.0)	48.0 (23.0, 135.0)		<0.001
ALT, U/L	54.0 (22.0, 177.0)		56.0 (23.0, 156.0)	50.0 (20.0, 195.8)		0.579
BUN, mmol/L	13.0 (9.0, 20.0)		14.0 (9.0, 22.0)	12 (9.0, 19.0)		<0.001
Creatinine, mg/dL	0.80 (0.60, 1.10)		0.80 (0.60, 1.20)	0.80 (0.70, 1.00)		0.762
Glucose, mg/dL	103.0 (87.0, 133.0)		106.0 (87.0, 139.0)	100.0 (86.0, 127.0)		0.001
Anion gap, mmol/L	14.0 (12.0, 16.0)		14.0 (12.0, 16.0)	14.0 (12.0, 16.0)		0.280
Bicarbonate, mmol/L	24.0 (22.0, 27.0)		24.0 (21.0, 26.0)	25.0 (23.0, 27.0)		<0.001
Sodium, mmol/L	139.0 (137.0, 141.0)		139.0 (136.0, 141.0)	139.0 (137.0, 141.0)		0.002
Potassium, mmol/L	3.90 (3.60, 4.30)		3.90 (3.50, 4.20)	4.00 (3.70, 4.30)		<0.001
Calcium, mmol/L	8.50 (8.10, 8.90)		8.10 (7.70, 8.30)	8.90 (8.70, 9.20)		<0.001
Length of stay, days	4.85 (2.91, 8.95)		5.81 (3.43, 11.49)	4.06 (2.72, 6.99)		<0.001
Hospital mortality, *n* (%)	115 (3.6)		83 (5.3)	32 (2)		<0.001

Continuous variables were presented as the median and interquartile range (IQR), and categorical variables were expressed as *n* (%). For categorical variables, *p* values were analyzed by *χ*^2^ test. For continuous variables, the Mann–Whitney *U* test was used in the nonnormal model. CHF : congestive heart failure, COPD : chronic obstructive pulmonary disease, CAD : coronary artery disease, CCI : Charlson comorbidity index, ICU : intensive care unit, SOFA : sequential organ failure assessment, SIRS : systemic inflammatory response system, SAPS : simplified acute physiology score, WBC : white blood cell count, TBil : total bilirubin, AST : aspartate aminotransferase, ALT : alanine aminotransferase, and BUN : blood urea nitrogen.

**Table 2:** Relative risk of having a hospital LOS of >2, >5, or >7 days was calculated according to the calcium level in different groups.

Characteristic	*N*	Univariate analysis		Model A		Model B		Model C	
		OR (95% CI)	*p* value	aOR (95% CI)	*p* value	aOR (95% CI)	*p* value	aOR (95% CI)	*p* value
LOS > 2 days									
Calcium, mg/dL			**<0.001**		**<0.001**		**<0.001**		**0.001**
<8.5	1580	1.00(ref)		1.00(ref)		1.00(ref)		1.00(ref)	
≥8.5	1576	**0.619(0.496, 0.772)**	**<0.001**	**0.623(0.499, 0.778)**	**<0.001**	**0.612(0.490, 0.765)**	**<0.001**	**0.653(0.507, 0.842)**	**0.001**
LOS > 5 days									
Calcium, mg/dL			**<0.001**		**<0.001**		**<0.001**		**<0.001**
<8.5	1580	1.00(ref)		1.00(ref)		1.00(ref)		1.00(ref)	
≥8.5	1576	**0.522(0.453, 0.601)**	**<0.001**	**0.525(0.456, 0.606)**	**<0.001**	**0.518(0.448, 0.597)**	**<0.001**	**0.589(0.503, 0.689)**	**<0.001**
LOS > 7 days									
Calcium, mg/dL			**<0.001**		**<0.001**		**<0.001**		**<0.001**
<8.5	1580	1.00(ref)		1.00(ref)		1.00(ref)		1.00(ref)	
≥8.5	1576	**0.468(0.402, 0.545)**	**<0.001**	**0.468(0.402, 0.546)**	**<0.001**	**0.463(0.397, 0.541)**	**<0.001**	**0.515(0.437, 0.609)**	**<0.001**

Adjusted covariates: model A: age, gender, race, marital status, insurance; model B: model A plus comorbidities; model: model B plus WBC, albumin, TBil, BUN, glucose, bicarbonate, sodium, and potassium. LOS : length of stay; CI: confidence interval; aOR: adjusted odds ratio; WBC : white blood cell count; TBil : total bilirubin; BUN : blood urea nitrogen. *p* value <0.05 is shown in bold.

## Data Availability

The data were obtained from the MIMIC-III public database (https://mimic.mit.edu). Everyone can request access to the data after completing the ethics test.
